# Curcumin inhibits proliferation, migration, invasion and promotes apoptosis of retinoblastoma cell lines through modulation of miR-99a and JAK/STAT pathway

**DOI:** 10.1186/s12885-018-5130-y

**Published:** 2018-12-10

**Authors:** Yaping Li, Weixuan Sun, Ning Han, Ying Zou, Dexin Yin

**Affiliations:** 1 Department of Ophthalmology, The Second Hospital of Jilin University, Changchun, Jilin, 130041 China; 2 Department of Gastroenterological Surgery, China-Japan Union Hospital of Jilin University, Changchun, Jilin, 130033 China; 3 Department of Vascular Surgery, China-Japan Union Hospital of Jilin University, No.126, Xiantai Street, Changchun, Jilin, 130033 China

**Keywords:** Curcumin, Retinoblastoma, miR-99a, JAK/STAT pathway

## Abstract

**Background:**

Curcumin, a primary active ingredient extracted from the *Curcuma longa*, has been recently identified as a potential anti-tumor agent in multiple kinds of cancers. However, the effect of curcumin on retinoblastoma (Rb) is still unclear. Therefore, we attempted to reveal the functional impacts and the underlying mechanisms of curcumin in Rb cells.

**Methods:**

Two Rb cell lines SO-Rb50 and Y79 were pre-treated with various doses of curcumin, and then cell proliferation, apoptosis, migration, and invasion were assessed, respectively. Further, regulatory effects of curcumin on miR-99a expression, as well as the activation of JAK/STAT pathway were studied.

**Results:**

Data showed that curcumin significantly inhibited the viability, colony formation capacity, migration and invasion, while induced apoptosis of SO-Rb50 and Y79 cells. Up-regulation of miR-99a was observed in curcumin-treated cells. Curcumin suppressed the phosphorylation levels of JAK1, STAT1, and STAT3, while curcumin did not inhibit the activation of JAK/STAT pathway when miR-99a was knocked down.

**Conclusion:**

Curcumin inhibited proliferation, migration, invasion, but promoted apoptosis of Rb cells. The anti-tumor activities of curcumin on Rb cells appeared to be via up-regulation of miR-99a, and thereby inhibition of JAK/STAT pathway.

## Background

Retinoblastoma (Rb) is a common malignant intraocular tumor among children [1], accounting for approximately 4% of all pediatric malignancies [2]. Orally chemotherapy alone failed to cure patients with intraocular Rb [3], while combination therapy, such as chemotherapy combined with focal therapy, has become the treatment of choice for intraocular Rb and with high cure rate [4]. Although the overall survival rates have been significantly improved recently, the survival rate of Rb in the developing nations is still unsatisfactory. The mainstay of therapy is for globe salvage.

Curcumin, a nature yellow pigment, is the primary active ingredient extracted from the rhizome of the East Indian plant *Curcuma longa* [5]. Currently, multiple therapeutic properties of curcumin have been recognized, including anti-inflammatory, anti-neoplastic [6], anti-oxidant [7], anti-fibrotic [8], and anti-ischemic [9] effects. Specifically regarding the anti-neoplastic function, curcumin has been reported to suppress the secretion of gastrin-mediated acid, and thereby inhibiting the progression of gastric cancer [10]. In vitro investigation has showed that curcumin inhibited bladder cancer cells growth and metastasis via regulating β-catenin expression [11]. Another study demonstrated that curcumin enhanced the radiosensitivity of renal cancer cells, suggesting the potential application of curcumin as an adjuvant in radiotherapy of renal cancer [12]. Although the anti-tumor potentials of curcumin in multiple kinds of cancers has been studied [13], the role of curcumin in Rb has not been well recognized.

Recent evidence has suggested that microRNA (miRNA) regulation is implicated in the anti-tumor properties of curcumin [14–16]. miRNAs are a class of short, non-coding RNAs that play significant roles in modulating various diseases progression. It has been reported that, miR-99a was frequently dysregulated in several human cancers, including breast cancer, nasopharyngeal carcinoma, esophageal squamous cell carcinoma and oral carcinoma, and the tumor-suppressive effects of miR-99a in these tumors have been revealed [17–20]. To date, no literature has focused on the tumor suppressive activities of miR-99a in Rb. Besides, a growing number of literatures have showed that, curcumin exerts its therapeutic properties through regulating the expression of cancer-related miRNAs [21, 22]. Therefore, herein we aimed to explore whether curcumin-mediated anti-tumor activity in Rb cells via modulation of miR-99a.

To this end, two Rb cell lines SO-Rb50 and Y79 were pre-treated with curcumin, and then cell growth and metastasis were evaluated, respectively. Further, the regulatory effects of curcumin on miR-99a expression, and JAK/STAT pathway were studied to explore the possible molecular mechanisms governing this tumor suppressive activity.

## Methods

### Cell lines and curcumin treatment

Rb cell lines, i.e., Y79 and SO-Rb50, were respectively obtained from the American Type Culture Collection (Catalogue number: ATCC® HTB-18, ATCC, Manassas, VA) and the Ophthalmic Center of Sun Yat-sen University (Guangzhou, China). The base medium for both Y79 and SO-Rb50 cell lines was RPMI-1640 medium (Life Technologies Corporation, Cergy Pontoise, France). To make the complete growth medium, 15% fetal bovine serum (FBS, Life Technologies Corporation), 0.1% ciprofloxacin, 2 mM L-glutamine, 1 mM sodium pyruvate, and 4.5% dextrose were added. Culture conditions were 37 °C in a humidified air with 5% CO_2_.

Curcumin with purity greater than 98% (Sigma-Aldrich, St. Louis, MO) was dissolved in dimethyl sulfoxide (DMSO, Sigma-Aldrich) at a concentration of 50 mM for stocking. The stock solution of curcumin was diluted by the culture medium so that the vehicle was less than 0.1%. Curcumin was used at concentration of 0–50 μM for 24 h.

### Cell viability

SO-Rb50 and Y79 cells (5 × 10^3^ cells/well) were planted in 96-well plated for 24 h of incubation. Thereafter, 0–50 μM of curcumin was added to treat cells for 24 h. Cell Counting Kit-8 (CCK-8, Dojindo Molecular Technologies, Gaithersburg, MD) solution (10 μL) was then added, and the cultures were incubated at 37 °C for another 2 h. The optical density was detected at 450 nm using the iMark microplate reader (Bio-Rad, Hercules, CA).

### Colony formation

SO-Rb50 and Y79 cells (500 cells/well) were seeded in 6-well plates. After adherence and curcumin treatment, the culture medium was replaced and the cells were cultured in normal medium for another two weeks. The colonies were fixed with 100% methanol and stained with 1% crystal violet (Sigma-Aldrich). Colonies containing more than 50 cells were defined as survivors.

### Apoptosis assay

FITC-annexin V/PI detection kit (Beijing Biosea Biotechnology, Beijing, China) was used in this study to quantify apoptotic cell rate after curcumin treatment. In brief, SO-Rb50 and Y79 cells (5 × 10^5^ cells/well) were planted in 6-well plates at. When cells were grown to about 80% confluence, cells were treated with 30 μM curcumin for 24 h. Thereafter, cells were collected, washed twice in PBS, resuspended in 200 μL binding buffer, and stained by 10 μL FITC-annexin V and 5 μL PI in the dark at room temperature for 30 min. Following the adding of 200 μL PBS, the fluorescence intensity was measured by a FACS scan (Beckman Coulter, Fullerton, CA).

### Transwell assay

A modified Boyden chamber with 8.0-μm pore filters (Costar-Corning, New York) was utilized in this study to evaluate cell migratory capacity following curcumin treatment. Cell invasion was carried out the same as migration assay, except that the transwell inserts were pre-coated with matrigel before assay. In brief, cells pretreated with 30 μM curcumin were suspended in 200 μL of serum-free medium. The cell suspension was added into the upper chamber of the 24-well plates, and 600 μL complete medium was added into the lower chamber. After incubation at 37 °C for 24 h, non-transferred cells were wiped off by cotton swabs. Transferred cells were stained with crystal violet and counted directly.

### miRNA transfection

miR-99a inhibitor with sequences of CACAAGAUCGGAUCUACGGGUU and its scrambled control (NC) were both purchased from GenePharma (Shanghai, China). Lipofectamine 3000 reagent (Invitrogen) was used for transfection following the manufacturer’s protocol. 48 h later, transfection was stopped and the efficiency of transfection was quantified by western blot.

### qRT-PCR

Cellular RNA was extracted using Trizol reagent (Life Technologies Corporation). RNA (5 μg) from each sample was subjected to reverse transcription using the Taqman MicroRNA Reverse Transcription Kit (Applied Biosystems, Foster City, CA). Taqman Universal Master Mix II was used in real-time PCR and each real-time PCR was carried out in triplicate for a total of 20 μL reaction mixtures on ABI PRISM 7500 Real-time PCR System (Applied Biosystems). Relative expression of CyclinD1 and miR-99a was normalized to GAPDH and U6 snRNA, respectively. The primers were as follows: CyclinD1, forward, 5′-TCC TCT CCA AAA TGC CAG AG-3′, and reverse, 5′-GGC GGA TTG GAA ATG AAC TT-3′; miR-99a, forward, 5′-GTT GGA TCC TAT TAA TAG GGG GCC CAT GCA AGA T-3′, reverse, 5′-GTT CTC GAG GCA CTG TGT ATA GCA TTT TGT CAG-3′.

### Western blot

Cellular proteins were extracted in 1% Triton X-100 and 1 mM PMSF (pH 7.4) over ice for 30 min. The extracts were centrifuged at 1200 *g* for 15 min at 4 °C and the supernatant were collected. Protein concentrations were quantified using the BCA™ Protein Assay Kit (Pierce, Appleton, WI). Protein (0.1 mg) was resolved over SDS-PAGE and transferred to a polyvinylidene fluoride membrane. The membranes were blocked in 5% non-fat dry milk for 1 h at room temperature, followed by probing with primary antibodies at 4 °C overnight: CyclinD1 (1:10000, ab134175), p21 (1:50, ab107099), Bcl-2 (1:500, ab59348), Bax (1:1000, ab199677), caspase-3 (1:250, ab13586), caspase-9 (1:200, ab25758), MMP2 (1:1000, ab37150), RhoA (1:5000, ab187027), ROCK1 (1:2000, ab45171), Vimentin (1:500, ab137321), JAK1 (1:300, ab125051), p-JAK1 (1:1000, ab215338), STAT1 (1:500, ab3987), p-STAT1 (1:1000, ab109461), STAT3 (1:500, ab119352), p-STAT3 (1:1000, ab30647), and β-actin (1:1000, ab8224, all from Abcam, Cambridge, MA). After incubation with the secondary antibodies, blots were visualized by enhanced chemiluminescence (ECL) method. Intensity of the positive blots was tested by Image Lab™ Software (Bio-Rad, Hercules, CA).

### Statistical analysis

Data were presented as mean ± standard derivations from three independent experiments. Statistical differences between two groups were analyzed using the Student *t* test, and between three or more groups were analyzed using the one-way analysis of variance (ANOVA). The SPSS version 13.0 software (SPSS Inc., Chicago, IL) was used to analyze statistical significance. A *P*-value of < 0.05 was considered to indicate a statistically significant result.

## Results

### Curcumin inhibited the proliferation of SO-Rb50 and Y79 cells

To start with, SO-Rb50 and Y79 cells were subjected with 0–50 μM of curcumin, and then the viability of cell was tested after 24 h treatment with curcumin. As a result, curcumin significantly reduced the viability of SO-Rb50 and Y79 cells (*P* < 0.05 or *P* < 0.01; Fig. 1a) in a dose-dependent manner. The IC50 values of curcumin in SO-Rb50 and Y79 cells were 38.4 and 34.8 μM, respectively. Thus, 30 μM was selected for use in the follow-up experiments. Results in Fig. 1b displayed that curcumin significantly reduced the survival rate of Rb cells (*P* < 0.001). Further results showed that curcumin down-regulated the expression of CyclinD1, while up-regulated the expression of p21 (*P* < 0.05 or *P* < 0.01; Fig. 1c and d). All these data provided the evidence that curcumin exerted anti-proliferating functions on Rb cells.

**Fig. 1:** Curcumin inhibited SO-Rb50 and Y79 cells proliferation. **a** Viability of cell pre-treated with 0–50 μM curcumin. **b** Colony formation capacity of cell pre-treated with 30 μM curcumin. **c** mRNA level expression of CyclinD1 in cell pre-treated with 30 μM curcumin. **d** Protein level expression of CyclinD1 and p21 in cell pre-treated with 30 μM curcumin. * *P* < 0.05, ** *P* < 0.01, *** *P* < 0.001 vs. control group

### Curcumin induced apoptosis in SO-Rb50 and Y79 cells

Impacts of curcumin on SO-Rb50 and Y79 cells apoptosis were determined. Results in Fig. 2a showed that, apoptotic cell rate was increased by addition of curcumin in both SO-Rb50 and Y79 cells (*P* < 0.01). Then, western blot analysis was carried out to determine the regulatory role of curcumin in apoptosis-related protein expression. Results in Fig. 2b and c displayed that, the ratio of Bcl-2 to Bax was significantly declined (*P* < 0.001), and caspase-3 and -9 were significantly cleaved (*P* < 0.001) in curcumin-treated cells. Thus, these results suggested the pro-apoptotic effects of curcumin on Rb cells.

**Fig. 2:** Curcumin promoted apoptosis in SO-Rb50 and Y79 cells. **a** Apoptotic cell rate of cell pre-treated with 30 μM curcumin. **b** Protein expression levels of apoptosis-associated factors in cell pre-treated with 30 μM curcumin. **c** Quantitative protein levels. ** *P* < 0.01, *** *P* < 0.001 vs. control group

### Curcumin inhibited the migratory and invasive capacities of SO-Rb50 and Y79 cells

Next, transwell assay was performed to ask whether curcumin also could affect SO-Rb50 and Y79 cells migration and invasion. Data in Fig. 3a and b revealed that, relative migration and invasion of SO-Rb50 and Y79 cells were both reduced by curcumin (*P* < 0.05 or *P* < 0.01). Results in Fig. 3c-e revealed that, the protein levels of MMP2, RhoA, ROCK1, and Vimentin were all down-regulated by curcumin (*P* < 0.05 or *P* < 0.01), which further confirmed the inhibitory role of curcumin in Rb cells migration and invasion.

**Fig. 3:** Curcumin inhibited the migratory and invasive capacities of SO-Rb50 and Y79 cells. **a** Relative migration and (**b**) relative invasion of cell after treatment with 30 μM curcumin. **c** and **d** Protein expression levels of metastasis-related factors in cell pre-treated with 30 μM curcumin. **e** Quantitative protein levels. * *P* < 0.05, ** *P* < 0.01 vs. control group

### Curcumin deactivated JAK/STAT signaling pathway via regulating miR-99a

Previous studies suggested that curcumin rendered its anti-tumor activities via regulating several miRNAs [14–16]. The present work attempted to study if miR-99a was a downstream gene of curcumin. The expression levels of miR-99a in cells pre-treated with or without curcumin were detected. qRT-PCR data showed that, miR-99a was up-regulated in cells treated with curcumin as relative to control cells (without curcumin treatment) (*P* < 0.05, Fig. 4a), which indicated that curcumin could efficiently up-regulate miR-99a expression in Rb cells. Then, miR-99a expression in SO-Rb50 and Y79 cells were suppressed by transfection with miR-99a inhibitor, to further explore whether the anti-tumor activity of curcumin was through enhancing miR-99a expression. Results in Fig. 4b showed that, miR-99a expression in cells transfected with miR-99a inhibitor was much lower than that in NC-transfected cells (*P* < 0.01), implying miR-99a-silenced cells were successfully established.

**Fig. 4:** Curcumin deactivated JAK/STAT signaling pathway. **a** miR-99a expression in cell pre-treated with 30 μM curcumin. **b** miR-99a expression in cell transfected with miR-99a inhibitor and NC. U6 snRNA was used as an internal control. **c** Protein expression levels of main factors in JAK/STAT pathway, after treatment with curcumin with or without miR-99a inhibitor transfection. **d** Quantitative protein levels. * *P* < 0.05, ** *P* < 0.01, *** *P* < 0.001 vs. control or NC groups. ## *P* < 0.01, ### *P* < 0.001 vs. curcumin + NC group

Several studies have suggested that curcumin exerted anti-inflammatory and anti-tumor effects through inhibiting JAK/STAT signaling pathway [23–28]. Herein, we explored whether miR-99a was implicated in the regulatory effect of curcumin on JAK/STAT pathway. Results showed that curcumin remarkably reduced the phosphorylation levels of JAK1, STAT1, and STAT3 (*P* < 0.05, *P* < 0.01 or *P* < 0.001). However, curcumin did not inhibit the phosphorylation of these proteins when miR-99a was knocked down (Fig. 4c and d).

## Discussion

Curcumin has been considered as a promising approach for the treatment of multiple cancers, including gastric cancer, bladder cancer, renal cancer, *etc* [6, 10–13]. Recently, several researchers also focused on the potential role of curcumin in Rb. Sreenivasan and his colleagues have reported that curcumin suppressed the expression of multidrug resistance associated protein 1 (MDR1) [29], thereby rendering Rb cells more sensitive to chemotherapy [30]. Another investigation demonstrated that curcumin induced the apoptosis of Y79 cells possibly through activating JNK and p38 MAPK pathways [31]. Although these authors have identified some anti-tumor activities of curcumin on Rb, additional studies are required to cross-check the anti-tumor properties of curcumin on other Rb cell types, and to decode the underlying mechanisms. Herein, we demonstrated that curcumin significantly inhibited the viability, colony formation capacity, migration and invasion of SO-Rb50 and Y79 cells, while curcumin could induce cell apoptosis to some extent. Furthermore, miR-99a was highly expressed in curcumin-treated cells. Curcumin could not block the activation of JAK/STAT signaling pathway when miR-99a was knocked down.

Previous studies showed that the anti-tumor activities of curcumin are mainly due to the inhibition of proliferation, migration and invasion, as well as due to the induction of apoptosis [11, 15, 22]. This study revealed that curcumin significantly reduced the viability and colony formation of both SO-Rb50 and Y79 cells, and the IC50 value of curcumin in these two Rb cell lines is about 35 μM. Besides, based on the data in the current study we inferred that curcumin-suppressed Rb cells proliferation might be via modulation of cell cycle, as CyclinD1 was down-regulated and p21 was up-regulated by addition of curcumin. Similar finding was reported by Yu et al. [31] that curcumin induced G1 phase arrest via down-regulations of Cyclin D3, CDK2/6, and up-regulations of p21 and p27. CyclinD1 and p21 are two key molecules in cell-cycle progression. CyclinD1 accelerates the G1/S transition, and p21 prevents cell cycle progression from the G1 to the S phase [32–34]. In addition to inhibiting Rb cells proliferation, we also demonstrated that curcumin was able to induce apoptosis, as apoptotic cell rate was increased, anti-apoptotic protein Bcl-2 was down-regulated, pro-apoptotic protein Bax was up-regulated, and caspase-3 and -9 were cleaved in curcumin-treated cells.

The occurrence of distant metastasis and organ infiltration [35] may lead to poor Rb prognosis. MMP2 is highly expressed in Rb [36], and pharmacological inhibition of MMP2 reduces Rb cells migration [37]. ROCK1 is a downstream effector of RhoA, RhoA/ROCK pathway is critical in controlling migration [38]. Vimentin is a well-known marker for epithelial-mesenchymal transition (EMT), which promotes cancer cells invasion and metastasis [39, 40]. Herein, data showed that curcumin reduced the relative migration and invasion of SO-Rb50 and Y79 cells, and reduced the expression levels of MMP2, RhoA, ROCK1 and Vimentin, suggesting the anti-migrating and anti-invasive roles of curcumin in Rb cells.

It has been reported that curcumin exerted anti-tumor activities via modulation of various miRNAs, including miR-21 [14], miR-340 [15] and miR-98 [16]. Curcumin could alter the expression of many miRNAs in Y79 cells [41], which may contribute to its anti-tumor properties in Rb. Herein, we for the first time demonstrated that curcumin treatment up-regulated miR-99a expression. In combination with the viewpoint obtained from previous studies that miR-99a is a tumor-suppressive miRNA in multiple cancers [17–20], we inferred that curcumin mediated anti-tumor activity in Rb possibly via regulating miR-99a expression.

The JAK/STAT pathway is one of the important signaling pathways in modulating cell proliferation, differentiation, migration and apoptosis [42]. Recent discoveries suggested that mutated JAK proteins will be potent target for anti-tumor therapy [43]. In this study, curcumin suppressed the phosphorylation of JAK1, STAT1 and STAT3 in both SO-Rb50 and Y79 cells. These findings were consistent with previous studies that suggested the anti-tumor effect of curcumin is through inhibiting JAK/STAT signaling pathway [26–28]. We additionally found that curcumin could not block JAK/STAT pathway in miR-99a-silenced cells, implying curcumin inhibited JAK/STAT pathway in a miR-99a-dependent mechanism.

In this study, the IC50 values of curcumin in two Rb cell lines (SO-Rb50 and Y79) were 38.4 and 34.8 μM, respectively, and 30 μM curcumin exhibited excellent anti-tumor activities. Due to the extensive intestinal and hepatic metabolic biotransformation, curcumin given orally resulted in low serum levels of curcumin. The peak serum concentration after 8000 mg of curcumin was 1.77 ± 1.87 μM [44]. Thus, it seems to be unfeasible to achieve 30 μM in the clinical use by the systemic route. Other routes of delivery of curcumin for Rb, including intravenous, intra-arterial, periocular and intravitreal techniques may be possible to achieve such a high concentration in the vitreous or the retina. Clinical usage of curcumin should take into account the ocular toxicity, ocular penetration, and systemic toxicity of Rb.

Nowadays, extensive preclinical studies over the past several decades have demonstrated the anti-tumor activities of curcumin in human cancers [10–13]. These preclinical studies suggested the potential efficacy of curcumin in clinical trials. In clinical studies, curcumin has been used either alone or in combination with other agents such as quercetin and gemcitabine to prevent or treat cancers [45, 46]. Phase I/II clinical studies have been conducted using curcumin and found that curcumin was helpful for overcoming chemo-resistance [47]. Our study provided in vitro evidences that curcumin has anti-Rb activities. However, significant research including animal and clinical trials is warranted to better understand the clinical value of curcumin in the treatment of Rb.

## Conclusions

To sum up, this study illuminated that curcumin inhibited proliferation, migration, invasion, and induced apoptosis of Rb cells. The anti-tumor activities of curcumin on Rb cells appear to be via up-regulation of miR-99a, and thereby inhibition of JAK/STAT pathway.

## Abbreviations

ANOVA: Analysis of variance
CCK-8Cell: Cell Counting Kit-8
DMSO: Dimethyl sulfoxide
ECL: Enhanced chemiluminescence
FBS: Fetal bovine serum
miRNA: MicroRNA
Rb: Retinoblastoma
